The article "TPPU Downregulates Oxidative Stress Damage and Induces BDNF Expression in PC-12 Cells" was retracted in 2023. Reasons: unreliable results or conclusions; concerns about the data; concerns about the peer review; concerns about the citations.

# TPPU Downregulates Oxidative Stress Damage and Induces BDNF Expression in PC-12 Cells

**DOI:** 10.1155/2022/7083022

**Published:** 2022-07-13

**Authors:** Qiong Wu, Minlin Lin, Peng Wu, Chongyan Zhao, Shuang Yang, Haiying Yu, Wenjiao Xian, Jingfang Song

**Affiliations:** ^1^Department of Basic Medicine, Guangdong Jiangmen Chinese Medicine College, Jiangmen, Guangdong Province, China 529000; ^2^Department of General Surgery, Jiangmen Wuyi Hospital of TCM, Jiangmen, Guangdong Province, China 529000

## Abstract

**Objective:**

Ischemia-reperfusion is an ongoing clinical challenge that can lead to a series of pathological changes including oxidative stress. The inhibition of soluble epoxide hydrolase inhibitor (sEH) by 1-(1-propanoylpiperidin-4-yl)-3-[4-(trifluoromethoxy)phenyl]urea (TPPU) results in an anti-inflammatory, cardioprotective, and blood vessel growth-promoting effects. Therefore, this study focused on the protective effect of TPPU on a rat pheochromocytoma (PC-12) cell oxidative stress model induced by H_2_O_2_.

**Methods:**

CCK-8 and Hoechst 33342 were used to evaluate cell apoptosis and western blot to detect the apoptotic proteins and brain-derived neurotrophic factor (BDNF) expression.

**Result:**

The incubation with 100 *μ*M, 50 *μ*M, and 25 *μ*M TPPU significantly increased PC-12 cell viability. Epoxyeicosatrienoic acid (EET) pretreatment also protected PC-12 cells from oxidative stress. In addition, TPPU reduced caspase-3 and Bax expression and induced Bcl-2 expression, and EETs exerted the same effect on caspase-3 expression as TPPU. A positive relationship was found between TPPU or EET incubation and BDNF expression.

**Conclusion:**

These results revealed that TPPU reduced PC-12 cell oxidative stress injury induced by H_2_O_2_ and promoted BDNF expression.

## 1. Introduction

Stroke is a serious nervous system condition associated with high morbidity, disability, and mortality [1]. It is the second leading cause of death, and the most of the global stroke burden originated in low- and middle-income countries [2]. The main symptoms of stroke may include pain, depression, cognitive function, fatigue, and disability [3]. Most strokes are of an ischemic type [4], and the reestablishment of blood flow may induce ischemia-reperfusion injury [5]. One of the main damage of ischemia-reperfusion is oxidative stress, which may destroy the respiration chain and phosphorylation, causing cell apoptosis and pathological damage, ultimately impairing the neurological function and inducing neuronal death [6]. Currently, no effective therapy for ischemia-reperfusion injury is available. A large number of studies focused on the exploration of ischemic reperfusion injury in stroke, but only a few have successfully passed clinical trials [7, 8].

The article "TPPU Downregulates Oxidative Stress Damage and Induces BDNF Expression in PC-12 Cells" was retracted in 2023. Reasons: unreliable results or conclusions; concerns about the data; concerns about the peer review; concerns about the citations.

Arachidonic acid (AA) is an important component of the cell membrane and is metabolized in three pathways: cytochrome P450 (CYP), lipoxygenase (LOX), and cyclic oxygenase (COX). Epoxyeicosatrienoic acid (EET) is metabolized through the AA-CYP pathway. 5,6-EET, 8,9-EET, 11,12-EET, and 14,15-EET are four isomers of EET [9]. EETs have a variety of similar biological functions, such as anti-inflammatory, antiapoptosis, antiplatelet aggregation, and vasodilator effects [10]. Since EETs are mainly hydrolyzed by soluble epoxide hydrolase, soluble epoxide hydrolase inhibitor (sEHI) may enhance their biological effects. 1-(1-propanoylpiperidin-4-yl)-3-[4-(trifluoromethoxy)phenyl]urea (TPPU) is a type of sEHI that is widely used on sEH studies. TPPU alleviates neural damage in BCAS-induced cerebral hypoperfusion by the activation of neuregulin-1/ErbB4 signaling [11]. TPPU also mitigates inflammation and protects the blood-brain barrier against ischemic injury [12]. The inhibition of sEH by TPPU also protects neurons from ischemic injury by suppressing mitochondrial apoptosis [13]. Our previous study showed that the injection of TPPU into mice produces antidepressant effects [14]. Increasing TPPU or EET level in corticosterone-pretreated PC-12 cells also reduces the neurotoxicity caused by corticosterone [15]. However, the effect of TPPU on oxidative stress-induced damages remains unknown.

Brain-derived neurotrophic factor (BDNF) is a secreted protein that is composed of 119 amino acids and has a relative molecular mass of 12 000 [16]. It is mainly distributed in the central nervous system, and its functions include the regulation of the survival, differentiation, and regeneration of glial cells and neurons; the promotion of myelin formation, neuronal migration, and axon growth; and the protection of damaged neurons [17]. A lack of BDNF may cause neurological conditions such as Parkinson's disease, brain atrophy, depression, and Alzheimer's disease [18–20]. Oxidative stress may also decrease BDNF expression [21]. Our previous study showed that the antidepressant effect caused by TPPU is closely related to the increase in BDNF level [14]; TPPU also increases BDNF expression and protects PC-12 cells damaged by corticosterone [15].

PC-12 cell line represents a suitable cell line for studying nervous and mental system diseases and is widely used to study oxidative stress damage to cells [22]. This study evaluated the cell protective effect and mechanism of TPPU on PC-12 cell oxidative stress induced by H_2_O_2_. The related changes in BDNF expression were also assessed.

The article "TPPU Downregulates Oxidative Stress Damage and Induces BDNF Expression in PC-12 Cells" was retracted in 2023. Reasons: unreliable results or conclusions; concerns about the data; concerns about the peer review; concerns about the citations.

## 2. Materials and Methods

### 2.1. Materials and Chemicals

The Chinese Academy of Medical Sciences provided the PC-12 cells. TPPU, H_2_O_2,_ Hoechst 33342, and primary antibodies anti-Bcl-2 and anti-Bax were purchased from Sigma Aldrich (USA). The cell culture reagents were obtained from Invitrogen (USA). EETs were obtained from Cayman Chemical (USA). Cell-counting kit-8 was purchased from Dojindo Molecular Technologies Inc. (USA). Anticleaved Caspase-3 antibody was obtained from Cell Signaling (USA), antibodies against BDNF were purchased from Millipore, and anti-GAPDH was bought from Boster (China).

TPPU was dissolved in 40% polyethylene glycol 400 (PEG 400). EETs were dried and dissolved in 40% PEG 400, and H_2_O_2_ was dissolved in 40% PEG 400 to prepare the working solutions.

### 2.2. Cell Culture and Treatment

Cryopreserved PC-12 cells were removed from liquid nitrogen, thawed at room temperature, and dissolved in cell culture medium composed of 1% penicillin-streptomycin, 10% FBS, and 89% DMEM. Approximately 2 × 10^5^/ml PC-12 cells were seeded in a culture dish and incubated under 5% CO_2_ at 37°C. The cell culture medium was replaced every other day.

Only cells in the exponential growth phase were selected for all experiments. Pretreatment with TPPU or a single dose of 1 *μ*M EET for 24 h and a final concentration of 100 *μ*M of H_2_O_2_ were added. All experiments were performed after further incubation of 16 h.

### 2.3. Cell Viability Assay

The CCK-8 assay kit in 96-well cell plates was used to assess cell viability as previously described [23]. After the treatment of the cells, 5 *μ*l CCK-8 was added to each well, and the cells were incubated at 37°C for 2 h. The absorbance was measured at 450 nm in a microplate reader. All experiments were repeated three times.

### 2.4. Hoechst 33342 Staining

PC-12 cells were fixed with 4% paraformaldehyde for 20 min at 37°C. Next, the cells were washed, and Hoechst 33342 staining solution at a final concentration of 5 mg/ml was added. The slices were then kept in the dark at room temperature for 15 min. The staining solution was removed, and the slices were washed and sealed. Cells were identified as apoptotic if the nuclei were densely stained or fragmented under microscopy examination [15].

### 2.5. Protein Extraction and Western Blotting

The cell culture was washed with ice cool PBS, and the remaining cells were lysed with RIPA buffer containing 100 *μ*M phenylmethanesulfonyl fluoride (PMSF) on ice to extract the total protein. Next, the cells were scraped off using a scraper and centrifuged for 5 min at 12000 RPM and 4°C. The BCA Protein Assay Kit was used to measure protein concentration. The extracted protein samples were stored at –20°C.

The article "TPPU Downregulates Oxidative Stress Damage and Induces BDNF Expression in PC-12 Cells" was retracted in 2023. Reasons: unreliable results or conclusions; concerns about the data; concerns about the peer review; concerns about the citations.

A total of 20 *μ*g protein samples/lane were added to 2× loading buffer and boiled at 100°C for 10 min. The proteins were loaded into 10% SDS-PAGE gel and separated by electrophoresis. Subsequently, the proteins were transferred to a PVDF membrane, which was incubated with 5% nonfat milk for 1 h to block the nonspecific bindings. Next, the membrane was incubated with the primary antibody (1 : 1000) at 4°C overnight and then with the corresponding HRP-conjugated secondary antibody for 1 h at room temperature. ECL Prime reagents were used to detect specific protein bands. FluroChem™ SP software was used to quantify the proteins.

### 2.6. Statistical Analysis

Statistical analysis was performed using SPSS 20.0 software (IBM, USA), and the results were expressed as ${\bar{X}}_{\pm }$ SEM. Comparisons among different groups were performed using one-way analysis of variance (ANOVA), while the post hoc least significant difference (LSD) test was selected in case of homoscedasticity. A value of *p* < 0.05 was considered statistically significant.

## 3. Results

### 3.1. TPPU Enhances Cell Viability Decreased by H_2_O_2_-Induced Oxidative Cell Injury

The effect of TPPU on H_2_O_2_-induced oxidative cell injury was evaluated by the CCK-8 assay. Control cells were considered as 100% viable cells. The results showed that 100 *μ*M H_2_O_2_ decreased PC-12 viability to 62.9%, while 100, 50, and 25 *μ*M TPPU significantly increased PC-12 viability to 97.1%, 99.8%, and 97.0%, respectively. However, 12.5 *μ*M TPPU incubation showed no protective effect against oxidative cell injury (cell viability 62.2%; Figure 1(a)). The incubation with 100 *μ*M H_2_O_2_ caused chromosome aggregation in the nucleus and nuclear fragmentation, indicating apoptosis as shown by Hoechst 33342 staining. Notably, 100, 50, and 25 *μ*M TPPU incubation reversed cell apoptosis. Consistent with the CCK-8 results, 12.5 *μ*M TPPU coculture did not exerted any protective effect on PC-12 cells against oxidative injury (Figure 1(b)).

### 3.2. EETs Enhance Cell Viability Decreased by H_2_O_2_-Induced Cell Damage

Since TPPU is an sEH inhibitor, inhibition of sEH may increase EETs activity. Therefore, the effect of EETs was investigated to evaluate whether it had the same cell-protective effect as TPPU. One *μ*M of all EETs significantly increased the viability of H_2_O_2_-injured PC-12 cells to 76.9%, 85.0%, 78.0%, and 81.7%, respectively (Figure 2). These results indicate that EETs protected the cells from oxidative stress.

### 3.3. TPPU Exerts Antiapoptotic Effects on Oxidative Stress-Induced Cell Apoptosis

Cells were incubated with 25 *μ*M TPPU for 24 h, and the extracted proteins were analyzed by western blot. The results showed that Caspase-3 and Bax protein expression decreased after TPPU treatment, while that of Bcl-2 increased (Figure 3). These results suggested that TPPU had an antiapoptotic effect on H_2_O_2_-induced oxidative injury.

The article "TPPU Downregulates Oxidative Stress Damage and Induces BDNF Expression in PC-12 Cells" was retracted in 2023. Reasons: unreliable results or conclusions; concerns about the data; concerns about the peer review; concerns about the citations.

### 3.4. TPPU Reverses H_2_O_2_-Induced Downregulation of BDNF

Western blot analysis was performed to further investigate whether TPPU improved BDNF expression in H_2_O_2_-injured PC-12 cells. The results revealed that the incubation with 25 *μ*M TPPU reduced the downregulation of BDNF expression in H_2_O_2_-induced oxidative damage (Figure 4).

### 3.5. Effect of EETs on Caspase-3 and BDNF in H_2_O_2_-Induced PC-12 Cell Apoptosis

The effects of TPPU on apoptotic protein and BDNF are shown in Figures 4 and 5. Western blot analysis was performed to further explore the protective effect of EETs, and the results showed a similar trend as TPPU. Caspase-3 protein expression in the groups treated with 1 *μ*M EETs was significantly decreased compared to its expression in the H_2_O_2_ group, whereas BDNF protein expression was increased. These results suggested that EETs could also exert an antiapoptotic effect in H_2_O_2_-induced oxidative injury.

## 4. Discussion

To our knowledge, this is the first study on the protective effect of sEH inhibitors in H_2_O_2_-induced oxidative cell damage. This study investigated the effects of TPPU and EETs against apoptosis of PC-12 cell induced by H_2_O_2_-induced oxidative stress. In general, 100, 50, and 25 *μ*M TPPU or 1 *μ*M EETs enhanced PC-12 cell viability. TPPU and EETs decreased caspase-3 and Bax expression, producing an antiapoptotic effect in H_2_O_2_-induced cell apoptosis. TPPU and EETs also abolished H_2_O_2_-induced downregulation of BDNF.

Electron acceptors and reactive oxygen species (ROS) are increased in ischemia-reperfusion injury. ROS are chemically active oxygen molecules containing metabolites that include peroxyl radicals (HO_2_), hydroxyl radicals (OH•), superoxide anion (O2•^−^), and nonradicals (H_2_O_2_, hypochlorous acid, and ozone). The brain consumes 20% of the body's oxygen [24] and produces more ROS during ischemia-reperfusion injury than other organs. ROS have diverse effects including DNA oxidation, activation of redox-sensitive transcription factors, protein modifications, activation of protein kinases, lipid peroxidation, and the opening of the ion channels [25]. H_2_O_2_ is a particularly important ROS [26] because it can cross the cell membrane and produce an apoptotic effect [27].

Since EETs are sEH substrates, sEH inhibitors enhance the bioactivity of EETs [28]. The inhibition of sEH enzyme activity, or the increase of the EET level, may produce antioxidative effects in a variety of pathologies. The silencing of the sEH 2 gene activates the PI3K/Akt/GSD3*β* pathway in H_2_O_2_-induced damage [29]. Park and Poo (2021) reported that EETs attenuate cisplatin nephrotoxicity through the stabilization of the mitochondrial transmembrane potential and reduction of oxidative stress [30]. However, the effects of sEH inhibitors or EETs on H_2_O_2_-induced oxidative PC-12 cell apoptosis are unknown. Our findings suggested that TPPU significantly reduced cell apoptosis in H_2_O_2_-induced oxidative stress, revealing, at least in part, the cell-protective effect.

The article "TPPU Downregulates Oxidative Stress Damage and Induces BDNF Expression in PC-12 Cells" was retracted in 2023. Reasons: unreliable results or conclusions; concerns about the data; concerns about the peer review; concerns about the citations.

BDNF is a member of the neurotrophic family of proteins. It is extensively distributed in the mammalian central nervous system where it modulates brain development [31]. BDNF protects neurons from apoptosis *in vivo* [32] and *in vitro* [33] and is strongly beneficial for cerebral ischemic-reperfusion injury [34]. Our previous study revealed that TPPU exerts rapid antidepressant effects in male mice, which are blocked by the BDNF-trkB pathway antagonist K252a [14]. TPPU also protects PC-12 cells from corticosterone injury by modulating BDNF expression [15]. This investigation demonstrated that the sEH inhibitor and EETs promoted BDNF expression in oxidative stress-damaged PC-12 cells. The mechanism used by TPPU or EETs inducing the increase of BDNF after oxidative stress needs further study.

In conclusion, this study reported the protective effect of TPPU on H_2_O_2_-induced cell apoptosis by analyzing cell viability and apoptosis. Western blot revealed that the apoptotic proteins were regulated by TPPU, and both TPPU and EETs also upregulated BDNF expression. New insights for understanding the role of the sEH inhibitor on ischemia-reperfusion injury are provided by these findings. Thus, TPPU might be used as a preventive and therapeutic treatment for ischemia-reperfusion injury, although further basic and clinical research are needed.

## Figures and Tables

**Figure 1:** TPPU protected H_2_O_2_-injured PC-12 cells. (a) The CCK-8 assay was used to assess the effect of TPPU on H_2_O_2_-induced oxidative cell injury. (b) Hoechst 33342 staining was used to determine apoptotic cells. ^∗∗∗^*p* < 0.001 compared to H_2_O_2_; ^###^*p* < 0.001 compared to H_2_O_2_.

**Figure 2:** Effects of EETs on H_2_O_2_-induced cell damage. PC-12 cells were pretreated with EETs for 24 h, and H_2_O_2_ was subsequently added. ^∗∗^*p* < 0.01 compared to H_2_O_2_; ^##^*p* < 0.01 compared to H_2_O_2_; ^###^*p* < 0.001 compared to H_2_O_2_.

**Figure 3:** Western blot analysis of Caspase-3, Bcl-2, and Bax protein expression. (a) Protein expression after incubation with 25 *μ*M TPPU for 24 h. (b–d) Caspase-3, Bcl-2, and Bax protein concentration were measured. ^∗∗^*p* < 0.01 compared to H_2_O_2_. ^∗∗∗^*p* < 0.001 compared to H_2_O_2_. ^##^*p* < 0.01 compared to H_2_O_2_. ^###^*p* < 0.001 compared to H_2_O_2_.

The article "TPPU Downregulates Oxidative Stress Damage and Induces BDNF Expression in PC-12 Cells" was retracted in 2023. Reasons: unreliable results or conclusions; concerns about the data; concerns about the peer review; concerns about the citations.

**Figure 4:** TPPU reduced H_2_O_2_-induced downregulation of BDNF. (a) Western blot analysis of BDNF expression. (b) BDNF protein concentration was measured (*n* = 3). ^∗∗∗^*p* < 0.001 compared to H_2_O_2_. ^##^*p* < 0.01 compared to H_2_O_2_.

**Figure 5:** EETs reversed the downregulation of caspase-3 and promoted BDNF expression in H_2_O_2_-induced oxidative stress. (a) Western blot analysis of caspase-3 and BDNF expression. (b, c) quantification of caspase-3 and BDNF expression (*n* = 3). ^∗∗∗^*p* < 0.001 compared to H_2_O_2_. ^###^*p* < 0.001 compared to H_2_O_2_.

## Data Availability

The datasets used and analyzed during the current study are available from the corresponding author upon reasonable request.
